The article "Differential Effects of Lichens versus Liverworts Epiphylls on Host Leaf Traits in the Tropical Montane Rainforest, Hainan Island, China" was published in 2014. Journal: ScientificWorldJournal.

# Differential Effects of Lichens versus Liverworts Epiphylls on Host Leaf Traits in the Tropical Montane Rainforest, Hainan Island, China

**DOI:** 10.1155/2014/681369

**Published:** 2014-06-04

**Authors:** Lingyan Zhou, Fude Liu, Wenjie Yang, Hong Liu, Hongbo Shao, Zhongsheng Wang, Shuqing An

**Affiliations:** ^1^The Laboratory of Forest Ecology and Global Changes, School of Life Sciences, Nanjing University, Nanjing 210093, China; ^2^School of Environmental Science and Safety Engineering, Tianjin University of Technology, Tianjin 300384, China; ^3^Department of Environmental Studies, Florida International University, Miami, FL 33199, USA; ^4^Center for Tropical Plant Conservation, Fairchild Tropical Botanic Garden, Coral Gables, Miami, FL 33156, USA; ^5^Key Laboratory of Coastal Biology & Bioresources Utilization, Yantai Institute of Coastal Zone Research, Chinese Academy of Sciences (CAS), Yantai 264003, China

## Abstract

Epiphylls widely colonize vascular leaves in moist tropical forests. Understanding the effects of epiphylls on leaf traits of host plants is critical for understanding ecological function of epiphylls. A study was conducted in a rain forest to investigate leaf traits of the host plants *Photinia prunifolia* colonized with epiphyllous liverworts and foliicolous lichens as well as those of uncolonized leaves. Our results found that the colonization of lichens significantly decreased leaf water content (LWC), chlorophyll (Chl) a and a + b content, and Chl a/b of *P. prunifolia* but increased Chl b content, while that of liverworts did not affect them as a whole. The variations of net photosynthetic rates (*P*_*n*_) among host leaves colonized with different coverage of lichens before or after removal treatment (a treatment to remove epiphylls from leaf surface) were greater than that colonized with liverworts. The full cover of lichens induced an increase of light compensation point (LCP) by 21% and a decrease of light saturation point (LSP) by 54% for their host leaves, whereas that of liverworts displayed contrary effects. Compared with the colonization of liverworts, lichens exhibited more negative effects on the leaf traits of *P. prunifolia* in different stages of colonization. The results suggest that the responses of host leaf traits to epiphylls are affected by the epiphyllous groups and coverage, which are also crucial factors in assessing ecofunctions of epiphylls in tropical forests.

## 1. Introduction

Carbon (C) enters ecosystems via the process of photosynthesis, which is the most important exchange between ecosystems and the atmosphere [1]. Leaf traits link closely with the photosynthetic characteristics of leaves and affect the capability of plants to sequestrate C [2–4]. However, leaves of vascular plants are usually covered with epiphylls [5, 6] in humid understory of the tropical forests. For example, up to 40% of the leaf surface was covered by epiphylls in an Australia tropical rain forest [7]. Epiphylls are usually small cryptogams growing on the upper surfaces of the host leaves [8] and commonly consist of two dominant visible groups: epiphyllous liverworts and foliicolous lichens (referred to as liverworts and lichens) [9].

The occurrence of epiphylls would induce a series of significant ecological and evolutionary impacts on host plants [10–12] due to the physical separation of epiphylls between the leaf surface and the atmosphere. Therefore, any potential change in epiphyllous communities, including shifting of community compositions and alteration of total coverage [13, 14], may considerably affect leaf traits of host plants subsequently. In addition, compared with vascular plants, epiphylls are more sensitive to environmental changes owing to their particular structure and physiology [15–17]. Whether or not epiphylls exacerbate or mitigate the effects of climate change on host vascular plants is crucial for understanding ecological functions of epiphyllous communities in tropical forests.

Previous studies paid more attention to nitrogen (N) transfer between epiphylls and hosts [9, 18–22] due to the ability of N fixation of epiphylls [23]. However, how epiphylls affect leaf physiological traits is still unclear [13, 14]. Some research has found that epiphylls decreased light radiation and photosynthetic capability of host leaves [24–27], while some thought that the photoacclimation of host plants could offset the negative effects of epiphylls [10, 28, 29]. These inconsistencies may result from the diverse composition of epiphyllous communities and undefined succession stages of epiphyllous colonization [14]. For examples, the epiphyllous groups in Monge-Najera (1989) and Anthony et al. (2002) were liverworts and lichens, respectively [10, 30].

Communities dominated by lichens or liverworts may induce different effects on leaf traits of host plants due to their diverse structure characteristics [15] and distribution patterns on host leaves [14, 31]. In addition, the coverage of epiphylls generally varies largely from sporadic to full cover [25, 31] in the successive process of epiphyllous colonization [7, 13, 14], which may be also crucial in understanding the roles of epiphylls on hosts. Therefore, it is necessary to differentiate effects of liverworts and lichens on host plants to better understand the exact roles of epiphylls on their host plants.

The tropical Montane rain forests in Hainan Island are the largest and best preserved primary tropical forest in China. The forests harbor diverse epiphylls on the surface of host leaves in the understory. In this study, we studied the effects of liverworts versus lichens, with varying degrees of covers on their host tree species* Photinia prunifolia* in a tropical Montane forest in Hainan Island. We asked the following questions: (1) Does epiphyllous colonization affect host's leaf traits? (2) Do the effects of epiphyllous groups (liverworts versus lichens) on host's leaf traits vary. (3) How do their coverages affect the effects on host's leaf traits?

## 2. Materials and Methods

### 2.1. Study Site and Species

The study was conducted in a tropical Montane rain forest at the Jianfengling National Nature Reserve (JNNR) (18°23′–18°50′N, 108°46′–109°02′E), which is located in the southwest of Hainan Island, China. JNNR is dominated by tropical monsoon climate, with an average air temperature of 24.5°C, relative humidity of 88%, and annual sunshine of 1467 h [32]. Annual precipitation ranges from 1305 to 3662 mm with a distinct wet season (May to October) and a dry season (November to April) [32]. The monthly temperature and precipitation there had been described by Yang et al. [33]. Due to the humid environment, approximately up to 14.5% leaf area of plants in the understory was covered with epiphylls (average percentage of leaves with epiphylls × average coverage on leaves), in which more than 60 species of epiphyllous liverworts have been identified (unpublished data). In order to obtain a relatively consistent species composition in epiphyllous communities, we selected host plants within a plot with a diameter of 5 km.

We selected the vascular plants,* Photinia prunifolia* as host plants in this study for the following reasons. Firstly,* P. prunifolia* was a common species with epiphylls at the study site. Secondly, the average coverage of epiphylls on the mature leaves of* P. prunifolia* was about 31.3%, which was ideal for sampling purpose. Thirdly, it was easy to remove epiphylls from coriaceous leaves of* P. prunifolia* for manipulative treatment. Leaves with comparable sizes and locations on the branches were selected from a large number of labeled leaves, which had been selected out two years ago when they were tender leaves with no epiphylls. We excluded leaves covered with mixed epiphyllous community of liverworts and lichens to avoid the interaction effects of the two groups. The dominant species of lichens on the surface of* P. prunifolia* were* Porina chrysophora* and* P. atrocaerulea*, and the dominant liverworts were* Drepanolejeunea spicata*,* Radula acuminata*,* Colura acroloba,* and* Leptolejeunea maculata*.

### 2.2. Measurement

Using a plastic sheet marked with 2 × 2 mm^2^ grids we measured the coverage of epiphylls (comprised of liverworts or lichens) on leaf surface following methods specified in Roskoski (1981) [13]. The leaves with 0% coverage of epiphylls (uncolonized leaves) were used as the control groups to be compared with leaves colonized by liverworts or lichens. Leaves colonized with liverworts or lichens were divided into four subgroups according to levels of coverage: 25%, 50%, 75%, and 100% (±5% error), respectively. The following physical leaf traits were measured: leaf mass per area (LMA), leaf water content (LWC), and chlorophyll (Chl) content (a and b). We used the method by Linder (1974) and Arnon (1949) for pretreatment and measurement of Chl content, respectively [34, 35]. The contents of Chl a, b, a + b (mg g^−1^), and a/b ratios were calculated subsequently. Physical leaf trait measurements were replicated 5 times for each subgroup, one replication per tree.

Before sampling, photosynthetic light-response curves of these leaves were examined using the “Light Curve” automatic program in Li-6400 Portable Photosynthesis System (LI-COR, USA) with a 6400-02B Red/Blue light source chamber (2 × 3 cm). Leaves were allowed 10 min to acclimate the changes of light intensity before measurements, which were made following photosynthetic photon flux (PPF): 0, 10, 20, 50, 100, 200, 500, 1000, 1500, and 2000 *μ*mol m^−2^ s^−1^, during 9:00–12:00 a.m, when the ambient temperature was 20 ± 2°C and relative humidity ranged from 50% to 70%. Airflow rate was kept constant at 0.5 L min^−1^ with 380 ± 10 *μ*mol mol^−1^ CO_2_ concentrations during the measurement.

In order to determine whether impacts of epiphylls on leaves were temporary, epiphylls were removed from the surface of leaves after photosynthetic measurement using methods described by Eze and Berrie (1977) [36]. Light-response curves of postremoval leaves were measured using the same method two days later after the removal treatment (hereafter, preremoval and postremoval were referred to the photosynthetic traits of leaves covered with epiphylls and those of epiphylls were removed, resp.). These measurements were replicated on 4 leaves from different trees in each subgroup. Parameters of photosynthetic light-response curves, which included respiration rate (*R*), maximum net photosynthesis rate (*P*_max⁡_), light compensation point (LCP), and light saturation point (LSP) in preremoval and postremoval, were estimated by nonrectangular hyperbola model [37]:

(1) $$\begin{array}{c} A=\frac{\varphi Q+A_{\max}-\sqrt{{\left(\varphi Q+A_{\max}\right)}^{2}-4\varphi QkA_{\max}}}{2k}-R, \end{array}$$

where *A* is net photosynthetic rate, *φ* is apparent quantum efficiency, *Q* is photosynthetically active radiation, *A*_max⁡_ is maximum net photosynthetic rate, *k* is an angle of photosynthesis light curve, and *R* is a dark respiration rate.

### 2.3. Data Analysis

Differences of leaf traits among the five levels of coverage (0%, 25%, 50%, 75%, and 100%) were tested by Tukey's multiple comparison. Student's *t*-test was used to investigate the differences of leaf traits between leaves covered with liverworts and lichens. The differences of leaf traits in the same leaves between pre- and postremoval treatments were tested by Paired-Samples *t*-test. Differences of net photosynthetic rates among light-response curves were examined by nonparametric tests (K related samples test). Effects of epiphyllous groups (liverworts and lichens), coverage (0%, 25%, 50%, 75%, and 100%), and removing treatment on physical traits of* P. prunifolia* leaves were examined using two-way ANOVA or three-way ANOVA.

## 3. Results

### 3.1. Physical Leaf Traits of Host Leaves with Different Epiphylls

The colonization of liverworts did not significantly affect all leaf traits of host (i.e., leaf mass per area (LMA), leaf water content (LWC), chlorophyll content (Chl), and Chl a/b ratio) with increasing coverage from 25 to 100% compared to the control group (0% coverage, Figure 1). The colonization of lichens significantly decreased LMA only at full coverage (*≈*100%) compared to the control group, while it decreased Chl a and Chl a + b at almost all coverage from 25 to 100% except Chl a + b at full coverage (Figures 1(a), 1(c), and 1(e)). Lichens significantly decreased LWC and Chl a/b and increased Chl b with increasing coverage when its coverage was larger than 50% (Figures 1(b), 1(d), and 1(f)).

Leaves covered with liverworts exhibited a significantly lower LMA than that in leaves colonized with lichens at coverage of 50% and 75% but displayed a significantly higher one compared to that with lichens at fall coverage (Figure 1(a)). The Chl b of leaves colonized with 75%–100% liverworts was also significantly lower than that colonized with lichens (Figure 1(d)). However, the LWC and Chl a/b of leaves covered with liverworts were significantly higher than that with lichens when the coverage was larger than 50% (Figures 1(b) and 1(f)). The Chl a and Chl a + b of leaves colonized with liverworts were all significantly higher than these with lichens (Figures 1(c) and 1(e)). The interactions of the levels of epiphyllous coverage (0%, 25%, 50%, 75%, and 100%) and groups (liverworts and lichens) were all significant in LMA, LWC, Chl a, Chl b, and Chl a/b (*P* < 0.05) except Chl a + b (*F* = 1.32, *P* > 0.05), while the main effect of coverage's levels on Chl a + b was significant (*F* = 3.71, *P* < 0.05) (Table 1).

### 3.2. Leaf Photosynthesis in Pre- and Postremoval Treatments

Net photosynthetic rates (*P*_*n*_) of light-response curves increased from 0 to 500 umol photons m^−2^ s^−1^ and then reached a plateau (Figure 2). Except for the leaves colonized with 25% liverworts, other light-response curves of* P. prunifolia* leaves (including those colonized by liverworts and lichens) were all significantly different from those in the uncolonized leaves (*P* < 0.05). With increasing coverage of epiphylls, *P*_*n*_ continuously increased from 25% to 75% while it decreased at 100% coverage (Figures 2(a) and 2(c)). In postremoval, most curves in leaves colonized by liverworts previously were no longer different significantly (*P* > 0.05) from those in uncolonized leaves, except that in leaves with 100% liverworts previously (*P* = 0.041). In contrast, differences in *P*_*n*_ between postremoval leaves colonized by lichens previously and uncolonized leaves were smaller than those between preremoval and uncolonized leaves but were still statistically significant (*P* < 0.05) (Figures 2(b) and 2(d)).

Epiphylls showed a negligible effect on total respiration rate (*R*) of leaves colonized with epiphylls in preremoval (left panel, Figure 3(a)), but the treatment of removing epiphylls resulted in a significant variation of *R* in most leaves of* P. prunifolia*, particularly for those with 25%–75% liverworts exhibited significant higher *R* (*P* < 0.05) compared with uncolonized leaves. Leaves colonized with 100% lichens had a significantly higher *R* (*P* = 0.040) in postremoval compared with those in preremoval (right panel, Figure 3(a)). With the exception of that in coverage and removal, interactions among epiphyllous groups, coverage, and treatment of removal (removal) were all significant in *R* of* P. prunifolia* leaves (Table 2). Epiphyll colonization did not affect the maximum net photosynthesis rates (*P*_max⁡_) of host leaves in general (*P* > 0.05, Figure 3(b)), except that of leaves with 50% lichens in preremoval with a higher *P*_max⁡_ (*P* = 0.042), in spite of the corresponding photosynthetic photon flux for *P*_max⁡_ that was different (Figure 2). The interaction of coverage and removal was significant in *P*_max⁡_.

The leaves of* P. prunifolia* colonized with lichens exhibited a significant higher light compensation point (LCP) at 100% coverage (11.6 *μ*mol m^−2^s^−1^) than that of uncolonized leaves (7.6 *μ*mol m^−2^ s^−1^). In contrast, the LCP of leaves colonized with 100% liverworts exhibited a significant lower one contrarily (left panel, Figure 3(a)). The difference in LCP between leaves colonized with lichens and liverworts became significant when the coverage is large enough (75%–100%, *P* < 0.05). In contrast, it was only significant at full coverage of epiphylls after removal (*P* = 0.048). The interaction of epiphyllous groups and coverage was significant on LCP (Table 2).

In preremoval, the difference in light saturation point (LSP) between leaves colonized with lichens and liverworts was also significant when the coverage was 100%. Removing treatment expanded the difference between epiphyllous groups in postremoval at full coverage and exhibited contrary effects on LSP between leaves colonized with liverworts and lichens. In postremoval, the LSP of leaves colonized with liverworts previously increased with an increasing degree of coverage and was significantly different from the uncolonized leaves at 75% and 100% coverage (Figure 3(d)). Full coverage of lichens decreased LSP of leaves by 54%, while that of liverworts increased LSP of leaves by 43%. The interactions of epiphyllous groups and coverage, groups, and removal were significant in LSP of* P. prunifolia* leaves (Table 2).

## 4. Discussion

### 4.1. Effects of Epiphylls on the Physical Leaf Traits of* P. prunifolia*

In tropical rain forest, light is one of the most important limitation affecting plant growth [2], especially in the understory which received only 0.5%–5.0% of the sunlight [12]. Thus, the wide distribution of epiphylls may make the low-light condition worse for hosts there [10, 36]. Host leaves are assumed to modify a series of physical traits in some extent to acclimate the colonization of epiphylls [30]. As a composite parameter associated with a suite of structural traits, leaf mass per area (LMA) can be understood as an index of leaf-level cost for light interception of host leaves and an important indicator of plant strategies [38, 39]. In this study, colonization of liverworts did not induce significant changes in host's LMA overall, while leaves with full coverage of lichens exhibited the lowest LMA. In addition, the leaves colonized with liverworts exhibited a significantly lower LMA than that with lichens at coverage of 50% and 75%, respectively (Figure 1(a)). In general, leaves possessed a lower LMA adapted to the low-light condition much better than that with a higher one [40, 41]. Therefore, the host leaves covered with liverworts (50%–75%) may be more competitive than that with lichens, especially under the increased shading condition [16]. However, leaves colonized with 100% lichens decreased LMA significantly by 18.6% compared with that in uncovered leaves, which may be attributed to the decline of photosynthetic output in mesophyll tissue due to the dense coverage of lichens [12, 42].

Lichens colonization on leaves of* P. prunifolia* also displayed a significantly negative effect on leaf water content (LWC) when the coverage was larger than 50% (Figure 1(b)), while the colonization of liverworts exhibited no effect on host's LWC at any coverage. Although some epiphylls (including lichens and liverworts) growing between the cuticle and epidermis had been indicated to absorb water from their hosts during periods of drought [8, 12, 16], the LWC of host leaves would not decline significantly unless the water transport of host plants was depressed by colonization of epiphylls [43]. Although both lichens and liverworts are poikilohydric, the former are more likely to occur in dry habitat than the latter [44]. This physiological drought of host leaves resulted from lichens colonization that may make lichens more competitive over liverworts and accelerate the senescence of host leaves accordingly [8, 25]. Therefore, the lowest LWC of leaves colonized with 100% lichens also supported the assumption that the leaves colonized with full cover of lichens may be ready for shedding [45].

Changes of chlorophyll contents in host leaves in response to epiphyllous colonization are crucial topics related to the acclimation of hosts to epiphyllous colonization [36, 46, 47]. The colonization of lichens significantly decreased chlorophyll content (Chl) a, a + b, and a/b (Figures 1(c), 1(e), and 1(f)) but increased Chl b in host leaves of* P. prunifolia* (Figure 1(d)), while the colonization of liverworts induced no changes of them even at full coverage (Figures 1(c)–1(f)). Combined with the change in LMA, lichens' effect on total chlorophyll content (*μ*g Chl cm^2^) of* P. prunifolia* was comparable with the results from Anthony et al. (2002) [10]. Lichens colonized on the leaves commonly are thought to prefer the habitat with higher light relative to liverworts [48]. Their absorptance spectra were also demonstrated to be similar to those of host leaves [10, 16], while most epiphyllous liverworts possessed lower Chl a/b ratio with higher levels of Chl b, and were adapted to low-light intensities better than did lichens [44]. Therefore, relative to light competition between liverworts and host leaves, the light competition between lichens and hosts would be more significant, which thus induced more modification in host's chlorophyll, such as decreased Chl a/b (Figure 1(f)) [28, 29].

### 4.2. Effects of Epiphylls on Photosynthesis of Host Leaves

Because of the independent photosynthetic capacity of liverworts and photobionts from lichens [15, 16, 49], the coating of epiphylls had been considered widely to affect the photosynthetic efficiency of host leaves [10, 13, 36]. With the exception of leaves colonized with 25% liverworts and full epiphylls, rates of C assimilation per unit leaf area colonized with epiphylls were all higher than that in single uncovered leaves of* P. prunifolia* (Figures 2(a) and 2(c)). Combined with the well-known contribution of epiphylls for N-fixation for host leaves [9, 18, 22], the colonization of epiphylls may increase the photosynthetic efficiency in community level at some extent. Although there is a general perception that both lichens and liverworts have low photosynthetic rates compared to their host vascular plants [15], the larger diversity of photosynthetic rates (*P*_*n*_) induced by increasing of lichens coverage implied a relative higher rate of lichens compared with that of liverworts (Figures 2(a) and 2(c)).

However, the respiration rate (*R*) and maximum net photosynthesis rates (*P*_max⁡_) of leaves with coating of lichens and liverworts did not show the expected increase as their larger intragroup variance in the same level of coverage excepted for the larger *P*_max⁡_ in leaves covered with 50% lichens (Figures 3(a) and 3(b), left panels). This negligible contribution of epiphylls to total *R* and *P*_max⁡_ was similar with that of lichens on host plants (*Calamus australis*) in Anthony et al. (2002) [10]. The full coverage of both lichens and liverworts induced some interesting changes of light compensation point (LCP) and light saturation point (LSP) (Figures 3(c) and 3(d), left panels). The full coverage of lichens induced an increased LCP but a decreased LSP of* P. prunifolia* leaves, which was inconsistent with general traits of plants in shading condition [50, 51], whereas leaves covered with dense liverworts were characterized by a decreased LCP contrarily. The dense coverage of liverworts advanced their hosts' shade tolerance [52], but without any significant impacts on their physical leaf traits compared with that in uncolonized leaves (Figure 1).

By removing epiphylls on host leaves, the effects of epiphylls to light-response curves were eliminated in postremoval; however, remained differences among bare leaves colonized with lichens previously were still larger than that with liverworts previously (Figure 2). The progressive colonization of lichens leaded to more accumulated effects on their host's photosynthetic capacity, which may concurrently occur with lichen-induced changes of physical leaf traits we discussed above (Figure 1). However, the significant increases of respiration rate (*R*) in some leaves induced by removal treatment were unexpected (Figure 3(a), right panel). The removal of dense lichen-induced increment of *R* in bare leaves may be attributed to the relative larger leaf area (the same as the area of leaf chamber) disturbed by removal treatment [53]. Leaves colonized with full lichens and liverworts before still exhibited an increased and a decreased LCP, respectively, after removal treatment (Figure 3(c), right panel), which also demonstrated that the lower LCP in the latter was one of acclimated leaf traits but not the temporary contribution from liverworts [14, 22]. The effects of removal treatment on LSP in leaves with full epiphylls were contrarily between that with full lichens and liverworts (Figure 3(d), right panel). The decreased LSP (by lichens) may prevent their leaves from utilizing sunflecks, which are commonly higher irradiances and important sources of photosynthetic photon flux (PPF) in the understory of tropical forests, whereas the increased LSP (by liverworts) may advance this capability to absorb them [51, 54].

### 4.3. Advantage of Liverworts in Epiphyllous Community

The relations between liverworts and lichens on phyllosphere are known as competitions, in which liverworts are generally preponderant and overgrow its opponent (lichens) [14, 16, 55]. For the host plants (*P. prunifolia*) we selected in this study, lichens' colonization had induced much more negative impacts on their physical leaf traits (Figure 1) as well as correlated photosynthetic parameters (e.g., LCP and LSP, Figure 3) compared to that of liverworts. In long term coevolution between epiphylls and host plants, epiphyllous group (liverworts) exhibited less disadvantageous effects on hosts that may possess more predominance in epiphyllous community [14], unless environmental changes favoring lichens competition.

In epiphyllous community, liverworts commonly require more proportion of available water than lichens [12]. Thus once available water in environment decreased, excessive water loss during drought periods in the understory of tropical rain forest may depress the advantage of liverworts in the competition with lichens [16]. Increasing frequency of drought and duration of heat waves may similarly induce more wide distribution of lichens [56, 57]. Thereby, current structure of epiphyllous community, including ratios of liverworts and lichens and total coverage on vascular plants, may shift to some extent in responding to these new ratios of available water and energy [58].

## 5. Conclusion and Prospect

In this study, the effects of epiphylls on host plants were focused on aspects of physical and photosynthetic leaf traits. Lichens colonization (especially at full coverage) significantly decreased leaf water content (LWC), chlorophyll (Chl) a and a + b content, and Chl a/b of* P. prunifolia* but increased Chl b content, while liverworts did not affect them as a whole (Figure 1). The variations of photosynthetic rates (*P*_*n*_) among host leaves induced by lichens before or after removal treatment were all larger than liverworts (Figure 2). The full coverage of lichens even induced an increased LCP but a decreased LSP of* P. prunifolia* leaves, while that of liverworts exhibited a contrary effect. Our results suggested that the effects of epiphyllous communities dominated by lichens or liverworts on host leaves had differentiated effects. Compared with liverworts, lichens colonization exhibited more adverse effects on their host's leaf traits. The coverage of epiphylls is a critical factor for determining the roles of epiphylls for host leaves, after all the vital effects on hosts only occur at largest coverage.

In natural understory of tropical rain forest, with colonization of epiphylls on phyllosphere, some symbiotic organisms with epiphylls provide the host leaf protection against herbivores and pathogens as well as the newly fixed nitrogen. The exact relationship between epiphylls and host plants is much more complicated than the modification of leaf traits. Furthermore, the advantage of liverworts relative to lichens exhibited in affecting host's leaf traits may shift with current environmental changes, as their environmental sensitivity and ecological fragility. More studies are needed to examine the ecophysiology of epiphylls, particularly under the background of climate change.

## Figures and Tables

**Figure 1:** Physical leaf traits of* Photinia prunifolia* colonized with lichens and liverworts at different coverages (0%, 25%, 50%, 75%, and 100%). (a) Leaf mass per area (LMA) (g m^−2^), (b) leaf water content (LWC) (%), (c) concentration of chlorophyll a (Chl a) (mg g^−1^), (d) concentration of chlorophyll b (Chl b) (mg g^−1^), (e) concentration of chlorophyll a + b (Chl a + b) (mg g^−1^), and (f) chlorophyll a/b ratio (Chl a/b) (mean ± 1 SE) (*n* = 5). Different lowercase letters above the bars indicate the differences of physical leaf traits among leaves colonized with lichens; the symbol * indicates the difference between leaves colonized with liverworts and lichens (*P* < 0.05).

**Figure 2:** Photosynthetic light-response curves of leaves of* Photinia prunifolia* colonized with liverworts (a and b) or lichens (c and d), pre- (a and c) versus postremoval (b and d) (mean ± 1 SE) (*n* = 4).

**Figure 3:** Estimated photosynthetic parameters of* Photinia prunifolia* colonized with lichens and liverworts, pre- versus postremoval (mean ± 1 SE) (*n* = 4). (a) Respiration rate (*R*), (b) maximum rates of photosynthesis (*P*_max⁡_), (c) light compensation point (LCP), and (d) light saturation point (LSP). The symbol * indicates the difference of photosynthetic parameters between pre- and postremoval treatment; different small and capital letters near the bars indicate the differences among leaves with different coverage and between leaves colonized with liverworts and lichens (*P* < 0.05).

**Table 1:** Effects (*F* value) of epiphyllous coverage (coverage: 0%, 25%, 50%, 75%, and 100%) and epiphyllous groups (groups: liverworts and lichens) on the leaf traits: leaf mass per area (LMA), leaf water content (LWC), concentration of chlorophyll a (Chl a), Chl b, Chl a + b, and Chl a/b of *Photinia prunifolia* in JNNR.

	df	LMA	LWC	Chl a	Chl b	Chl a + b	Chl a/b
Coverage	4	8.62***	3.01*	4.98**	2.67*	3.71*	1.55^ns^
Groups	1	2.09^ns^	15.1***	30.9***	5.94*	3.52^ns^	19.0***
Coverage × groups	4	5.46**	3.17*	5.55**	3.03*	1.32^ns^	6.01**

*P < 0.05, **P < 0.01, ***P < 0.001, ^ns^Not significant.

**Table 2:** Effects of epiphyllous coverage (0%, 25%, 50%, 75%, and 100%), epiphyllous groups (groups: liverworts and lichens), and treatment of removal (preremoval and postremoval) on photosynthetic parameters: respiration rate (*R*), maximum rates of photosynthesis (*P*_max⁡_), light compensation point (LCP), and light saturation point (LSP) of *Photinia prunifolia* in JNNR.

Source	df	*R*	*P*_max⁡_	LCP	LSP
Groups	1	0.88^ns^	3.86^ns^	20.6***	16.0***
Coverage	4	1.68^ns^	18.5***	0.556^ns^	10.2***
Removal	1	8.46**	29.1***	0.120^ns^	1.14^ns^
Groups × coverage	4	2.90*	1.20^ns^	6.65***	18.6***
Coverage × removal	4	1.60^ns^	5.91***	0.566^ns^	2.32^ns^
Groups × removal	1	8.34**	2.15^ns^	1.15^ns^	6.49*
Groups × coverage × removal	4	5.70***	2.05^ns^	0.239^ns^	2.31^ns^

*P < 0.05, **P < 0.01, ***P < 0.001, ^ns^Not significant.

## References

[1] Lange OL, Beyschlag W, Tenhumen JD, Schulze ED, Zwlfer H (1987). Control of leaf carbon assimilation-input of chemical energy into ecosystems. *Potentials and Limiatations of Ecosystem Analysis*.

[2] Poorter L (1999). Growth responses of 15 rain-forest tree species to a light gradient: the relative importance of morphological and physiological traits. *Functional Ecology*.

[3] Rozendaal DMA, Hurtado V, Poorter L (2006). Plasticity in leaf traits of 38 tropical tree species in response to light; relationships with light demand and adult stature. *Functional Ecology*.

[4] Trewavas A (2009). What is plant behaviour?. *Plant, Cell and Environment*.

[5] Lücking R (1997). *Additions and Corrections to the Knowledge of the Foliicolous Lichen Flora of Costa Rica: The Family Gomphillaceae*.

[6] Lücking R (1999). Ecology of foliicolous lichens at the “Botarrama” trail (Costa Rica), a neotropical rainforest. IV. Species associations, their salient features and their dependence on environmental variables. *The Lichenologist*.

[7] Rogers JS, Clark E, Cirvilleri G, Lindow SE (1994). Cloning and characterization of genes conferring copper resistance in epiphytic ice nucleation-active Pseudomonas syringae strains. *Phytopathology*.

[8] Berrie GK, Eze JMO (1975). The relationship between an epiphyllous liverwort and host leaves. *Annals of Botany*.

[9] Bentley BL, Carpenter EJ (1984). Direct transfer of newly-fixed nitrogen from free-living epiphyllous microorganisms to their host plant. *Oecologia*.

[10] Anthony PA, Holtum JAM, Jackes BR (2002). Shade acclimation of rainforest leaves to colonization by lichens. *Functional Ecology*.

[11] Coley PD, Kursar TA, Mulkey SS, Chazdon RL, Smith AP (1996). Anti-herbivore defenses of young tropical leaves: physiological constraints and ecological trade-offs. *Tropical Forest Plant Ecophysiology*.

[12] Coley PD, Kursar TA, Machado JL (1993). Colonization of tropical rain-forest leaves by epiphylls—effects of site and host plant leaf lifetime. *Ecology*.

[13] Roskoski JP (1981). Epiphyll dynamics of a tropical understory. *Oikos*.

[14] Zhou L-Y, Wang Z-S, Chen S-N (2009). Advances in researches on ecological epiphylls. *Chinese Journal of Plant Ecology*.

[15] Green T, Lange O (1994). Photosynthesis in poikilohydric plants: a comparison of lichens and bryophytes. *Ecophysiology of Photosynthesis*.

[16] Pinokiyo A, Singh KP, Singh JS (2006). Leaf-colonizing lichens: their diversity, ecology and future prospects. *Current Science*.

[17] Pócs T (2009). Epiphyllous liverwort diversity at worldwide level and its threat and conservation. *Anales del Instituto de Biología Serie Botánica*.

[18] Bentley BL (1987). Nitrogen fixation by epiphylls in a tropical rainforest. *Annals of the Missouri Botanical Garden*.

[19] Bentley BL, Carpenter EJ (1980). Effects of desiccation and rehydration on nitrogen fixation by epiphylls in a tropical rainforest. *Microbial Ecology*.

[20] Freiberg E (1998). Microclimatic parameters influencing nitrogen fixation in the phyllosphere in a Costa Rican premontane rain forest. *Oecologia*.

[21] Palmqvist K, Dahlman L (2006). Responses of the green algal foliose lichen *Platismatia glauca* to increased nitrogen supply. *New Phytologist*.

[22] Wanek W, Pörtl K (2005). Phyllosphere nitrogen relations: reciprocal transfer of nitrogen between epiphyllous liverworts and host plants in the understorey of a lowland tropical wet forest in Costa Rica. *New Phytologist*.

[23] Roskoski JP (1980). N_2_ fixation (C_2_H_2_ reduction) by epiphylls on coffee, *Coffea arabica*. *Microbial Ecology*.

[24] Chazdon RL, Fetcher N (1984). Photosynthetic light environments in a lowland tropical rain forest in Costa Rica. *Journal of Ecology*.

[25] Clark DB, Clark DA, Grayum MH (1992). Leaf demography of a neotropical rain forest cycad, *Zamia skinneri* (Zamiaceae). *The American Journal of Botany*.

[26] Oberbauer SF, Clark DA, Clark DB, Quesada M (1989). Comparative-analysis of photosynthetic light environments within the crowns of juvenile rain-forest trees. *Tree Physiology*.

[27] Oberbauer SF, Clark DB, Quesada M (1988). Crown light environments of saplings of two species of rain forest emergent trees. *Oecologia*.

[28] Chazdon RL, Pearcy RW, Lee DW, Fetcher N, Mulkey SS, Chazdon RL, Smith AP (1996). Photosynthetic responses of tropical forest plants to contrasting light environments. *Tropical Forest Plant Ecophysiology*.

[29] Lambers H, Chapin FS, Pons TL (1998). *Plant Physiological Ecology*.

[30] Monge-Najera J (1989). The relationship of epiphyllous liverworts with leaf characteristics and light in Monte Verde, Costa Rica. *Cryptogamie, Bryologie*.

[31] Sonnleitner M, Dullinger S, Wanek W, Zechmeister H (2009). Microclimatic patterns correlate with the distribution of epiphyllous bryophytes in a tropical lowland rain forest in Costa Rica. *Journal of Tropical Ecology*.

[32] Zhou Z, Li Y-D, Lin M-X (2009). Change characteristics of thermal factors in tropical mountain rainforest area of Jianfen-gling, Hainan Island in 1980–2005. *Chinese Journal of Ecology*.

[33] Yang W, Liu F, Zhou L, Zhang S, An S (2013). Growth and photosynthetic responses of Canarium pimela and Nephelium topengii seedlings to a light gradient. *Agroforestry Systems*.

[34] Arnon DI (1949). Copper enzymes in isolated chloroplasts—polyphenoloxidase in beta-vulgaris. *Plant Physiology*.

[35] Linder S (1974). A proposal for the use of standardised methods for chlorophyll determination in ecological and ecophysiological investigations. *Physiologia Plantarum*.

[36] Eze JMO, Berrie GK (1977). Further investigations into the physiological relationship between an Epiphyllous Liverwort and its host leaves. *Annals of Botany*.

[37] Prioul JL, Chartier P (1977). Partitioning of transfer and carboxylation components of intracellular resistance to photosynthetic CO_2_ fixation: a critical analysis of the methods used. *Annals of Botany*.

[38] Klein I, Dejong TM, Weinbaum SA, Muraoka TT (1991). Specific leaf weight and nitrogen allocation responses to light exposure within Walnut trees. *Hortscience*.

[39] Poorter H, Niinemets Ü, Poorter L, Wright IJ, Villar R (2009). Causes and consequences of variation in leaf mass per area (LMA): a meta-analysis. *New Phytologist*.

[40] Niinemets Ü (1997). Role of foliar nitrogen in light harvesting and shade tolerance of four temperate deciduous woody species. *Functional Ecology*.

[41] Walters MB, Kruger EL, Reich PB (1993). Growth, biomass distribution and CO_2_ exchange of northern hardwood seedlings in high and low light: relationships with successional status and shade tolerance. *Oecologia*.

[42] Rogers RW, Barnes A (1986). Leaf demography of the rainforest shrub Wilkiea macrophylla and its implications for the ecology of foliicolous lichens. *Australian Journal of Ecology*.

[43] Ivey CT, Desilva N (2001). A test of the function of drip tips. *Biotropica*.

[44] Marschall M, Proctor MCF (2004). Are bryophytes shade plants? Photosynthetic light responses and proportions of chlorophyll a, chlorophyll b and total carotenoids. *Annals of Botany*.

[45] Richards PW (1952). *The Tropical Rain Forest: An Ecological Study*.

[46] Lücking R, Bernecker-Lücking A (2005). Drip-tips do not impair the development of epiphyllous rain-forest lichen communities. *Journal of Tropical Ecology*.

[47] Toomey M, Roberts D, Nelson B (2009). The influence of epiphylls on remote sensing of humid forests. *Remote Sensing of Environment*.

[48] Coley PD, Kursar TA, Mulkey SS, Chazdon RL, Smith AP (1996). Causes and consequences of epiphyll colonization. *Tropical Forest Plant Ecophysiology*.

[49] Zotz G, Winter K (1994). Photosynthesis and carbon gain of the lichen, Leptogium azureum, in a lowland tropical forest. *Flora*.

[50] Bohning R, Burnside CA (1956). The effect of light intensity on rate of apparent photosynthesis in leaves of sun and shade plants. *The American Journal of Botany*.

[51] Kitajima K (1994). Relative importance of photosynthetic traits and allocation patterns as correlates of seedling shade tolerance of 13 tropical trees. *Oecologia*.

[52] Craine JM, Reich PB (2005). Leaf-level light compensation points in shade-tolerant woody seedlings. *New Phytologist*.

[53] Ribas-Carbo M, Taylor NL, Giles L (2005). Effects of water stress on respiration in soybean leaves. *Plant Physiology*.

[54] Chazdon RL, Pearcy RW (1991). The importance of sunflecks for forest understory plants. *BioScience*.

[55] Olarinmoye S (1974). Ecology of epiphyllous liverworts: growth in three natural habitats in Western Nigeria. *Journal of Bryology*.

[56] Ellis CJ, Coppins BJ, Dawson TP (2007). Predicted response of the lichen epiphyte Lecanora populicola to climate change scenarios in a clean-air region of Northern Britain. *Biological Conservation*.

[57] Ellis CJ, Yahr R, Coppins BJ (2009). Local extent of old-growth woodland modifies epiphyte response to climate change. *Journal of Biogeography*.

[58] Stephenson NL (1990). Climatic control of vegetation distribution: the role of the water balance. *The American Naturalist*.

